# Evaluation of the Effect of *Lactobacillus acidophilus* ATCC 4356 Bacteriocin against *Staphylococcus aureus*

**DOI:** 10.1155/2024/4119960

**Published:** 2024-03-22

**Authors:** Zeinab Fagheei Aghmiyuni, Horieh Saderi, Parviz Owlia, Navid Saidi

**Affiliations:** Molecular Microbiology Research Center, Shahed University, Tehran, Iran

## Abstract

**Background:**

*Lactobacillus acidophilus* is lactic acid bacteria that produce bacteriocins. Bacteriocins are antimicrobial peptides or proteins that exhibit activity against closely related bacteria. The aim of this study was to determine the effect of *L. acidophilus* ATCC 4356 bacteriocin against *Staphylococcus aureus. Material and Methods*. We used four different phenotypic methods for antimicrobial activities against two standard strains: methicillin-resistant *S. aureus* (MRSA) ATCC 33591 and methicillin-susceptible *S. aureus* (MSSA) ATCC 25923. The methods were (1) agar well diffusion, (2) overlay soft agar, (3) paper disk, and (4) modification of punch hole. The ammonium sulfate method was used to concentrate crude bacteriocin, and ultrafiltration and dialysis tubes were used to remove ammonium sulfate from the bacteriocins. Each method was repeated in triplicate.

**Result:**

*L. acidophilus* ATCC 4356 showed antimicrobial activity against both MRSA and MSSA standard strains only by the overlay soft agar method and not by the agar well diffusion, punch hole modification, and paper disk methods. No antimicrobial effects were observed in crude bacteriocins concentrated.

**Conclusion:**

The growth inhibition of *S. aureus* in overlay soft agar method may be due to the production of bacteriocin-like substances. The overlay soft agar method is a qualitative test, so there is a need for further study to optimize the conditions for the production of bacteriocin-like substances in the culture supernatant and precise comparison between the inhibitory activity and pheromone secretion of different strains.

## 1. Introduction

*Staphylococcus aureus* (*S. aureus*) is a main human pathogen and causes a variety of infections and diseases including skin and soft tissue infections to severe and life-threatening systemic diseases such as endocarditis, osteomyelitis, and necrotizing fasciitis [1, 2]. *S. aureus* is the most important reason for nosocomial infections among antibiotic-resistant organisms [3]. The increase in multi-drug-resistant *S. aureus* strains has increased the rate of resistance to infection, thus making clinical anti-infective treatments more difficult. Methicillin-resistant *S. aureus* (MRSA) is a kind of multi-drug-resistant “super bacteria” resistant to *β*-lactam antibiotics and aminoglycosides, quinolones, and macrolides [4]. The rapid spread of multi-drug-resistant (MDR) pathogens has reduced the efficiency of common antibiotics. Diseases caused by MDR pathogens are a serious worldwide public health problem [5]. One of the world's most important infectious diseases due to its high morbidity and mortality is an infection caused by MRSA, which threatens human health and has concerned the responsiveness of the global medical community [4]. Therefore, finding and developing new antimicrobial agents and effective drugs to treat infections due to MDR bacteria are vital. Bacteriocins are the most important group of antimicrobial peptides (AMPs) with applications in human health [6]. Bacteriocins are produced by gram-positive (GPB) and gram-negative bacteria. The enormous majority of bacteriocins described are produced by GPB, especially lactic acid bacteria (LAB) including *lactobacilli*, *lactococci*, and *pediococci* [7]. The ability of bacteriocin production has been tested by biochemical and genetic studies, and they can be classified according to their biochemical and genetic characteristics [8, 9]. Bacteriocins are heat-stable, ribosomal-synthesized AMPs [8] and in GPB classified into three different groups: lantibiotics and nonlantibiotics of low and high molecular weight. Class I consist of lantibiotics, and they are small (<5 kDa) and heat-stable peptides that affect membrane structures. Class II consists of nonlantibiotics, and they have variable molecular weight but are usually small (<10 kDa) and heat-stable and contain regular amino acids. Class III of bacteriocins has large peptides (>30 kDa) and heat-labile antimicrobial proteins [10–12]. In recent years, antibiotic resistance in strains of *S. aureus* has developed and is a significant threat to humanity [13]. Therefore, bacteriocins produced by LAB isolates and applied as alternative antimicrobial compounds against pathogen bacteria are ideal candidates for this threat. The present study was aimed at assessing the antibacterial capacity of bacteriocin produced by *Lactobacillus acidophilus* ATCC 4356 against *Staphylococcus aureus.*

## 2. Materials and Methods

### 2.1. Strain and Culture Condition

*Lactobacillus acidophilus* (*L. acidophilus*) ATCC 4356 was purchased and lyophilized from Persian Type Culture Collection (PTCC), Culture and Research, Tehran, Iran. It was grown in Man-Rogosa-Sharpe broth (MRSB) and incubated at 37° C for 48 hours in an anaerobic jar and maintained on Man-Rogosa-Sharpe (MRS) agar. Methicillin-resistant *S. aureus* (MRSA) standard strains ATCC 33591 and methicillin-susceptible *S. aureus* (MSSA) ATCC 25923 were grown in separated plates of nutrient agar and incubated at 37°C for 18 hours in aerobic condition.

### 2.2. Antimicrobial Activity Assay

We used four methods for the preliminary investigation of antimicrobial activity against MRSA and MSSA. These methods are comprised of the solid culture method with overlay soft agar and liquid culture method with agar well diffusion, the paper disk method, and the modification of punch hole. Bacteriocin sensitivity was assessed as clear zones of growth inhibition surrounding the *L. acidophilus*.

#### 2.2.1. Overlay Soft Agar Method

The overlay soft agar or deferred method was done with the method of the agar spot test used by Hernández et al. with some modifications [14, 15]. A single colony of *L. acidophilus* ATCC 4356 was spotted on the MRS agar plates and incubated at 37°C in an anaerobic jar for 24 h (instead of dissolving MRS powder in distilled water, phosphate buffer saline (PBS) solution (0.05 M, pH = 7.4) was used). PBS was used to maintain the pH of the culture medium). After that, the lid of the plates was removed, and the agar plates were reversed on wet cotton with chloroform for 20 minutes (this was done to kill viable bacteria with chloroform vapor so that only extracellular products remained on the plate). Then, 50 *μ*l of overnight MRSA and MSSA standard strains was separately added to two tubes containing 5 ml soft BHI broth supplemented with 0.7% agar, mixed, poured onto the two plates, and incubated at 37°C for 24 h. In order to optimize the conditions for better bacteriocin production, this method was performed several times with changes in the incubation time including 18, 24, 48, and 72 hours.

#### 2.2.2. Agar Well Diffusion Method

Cell-free supernatant (CFS) was obtained by centrifugation of *L. acidophilus* culture in MRS broth at 4500 rpm for 10 min at 4°C. Then, the supernatant was sterilized by filtration through a 0.22 *μ*l syringe filter. The CFS was neutralized with sufficient amounts of 5 M NaOH to remove the possible antimicrobial effect of the organic acid (pH 6.5) and compared with unneutralized CFS. In this study, The CFS was not treated with catalase to eliminate the possible effect of H_2_O_2_, because *S. aureus* is a catalase-positive organism. This CFS was used for agar well diffusion and modification of punch hole methods.

The test organisms were inoculated in nutrient broth, and suspensions were prepared at a concentration to adjust the turbidity to 0.5 McFarland standards, giving a final inoculation of 1.5 × 10^8^ CFU/ml. Wells of 6 mm were bored in the inoculated media with the help of a sterile blue sampler tip (6 mm). Each well was filled with 100 *μ*l CFS and control sample: positive control (gentamicin disk 30 mcg) and negative control (PBS). It was allowed to diffuse for about 30 minutes at room temperature and incubated for 18–24 hours at 37°C. In order to optimize the conditions for better bacteriocin production, this method was performed several times with changes in TSB, BHI, MRS liquid culture media, and incubation temperatures of 30 and 37°C for 18, 24, 48, and 72 hours [16].

#### 2.2.3. The Paper Disk Method

The test organisms were grown at 37°C in 4 ml of tryptic soy broth (TSB) media. After overnight culture, all test organisms were smeared on tryptic soy agar (TSA) plates, and blank paper disks (6 mm) were placed on the plates, and then, 10 *μ*l of overnight-cultured broths of *L. acidophilus* in 4 ml of an MRS broth media containing 5% (*w*/*v*) NaCl was added onto the disks and plates incubated for 18–24 hours at 37°C. A gentamicin disk (30 mcg) was used for positive controls, and a MRS broth medium containing 5% (*w*/*v*) NaCl was used for negative control [17].

#### 2.2.4. Modification of Punch Hole Method

This procedure was performed according to the method described by Tagg and McGiven [18]. Petri dishes are filled with an appropriate nutrient medium to a thickness of 5 mm; various numbers of holes are punched out of the agar, by using a sterile blue sampler tip of 6 mm diameter. The base of each hole is sealed with a drop (0.05 ml) of melted nutrient agar, and CFS (1, 2, or 3 drops) of *L. acidophilus* preparations is added to the appropriate wells. The inoculated plates are incubated at 37°C for 1 to 2 h to allow for diffusion of the bacteriocin into the medium. The agar is then loosened from the edge of the petri dish with a sterile spatula; the medium were inverted and prized away from the dish so that it falls into the lid, exposing the bottom surface of the agar. After drying at 37°C for 2 h, the freshly exposed surface is inoculated by flooding with a log phase culture of the appropriate test organism. The plates are drained, dried, and then incubated for 18–24 hours at 37°C with lids uppermost until zones of inhibition have clearly developed.

### 2.3. Concentration of Crude Bacteriocins by Ammonium Sulfate Method

A 0.5 McFarland (1.5 × 10^8^ CFU/ml) suspension was prepared from *L. acidophilus*. Then, 5 ml of this suspension was inoculated into 100 ml of MRS and incubated for 24 h at 37°C and an optimal pH 6.2 in an anaerobic atmosphere. Culture broth media were adjusted to pH 6.2 by adding sufficient amounts of 1 N NaOH. The bacterial CFS was collected by centrifugation at 6,000 g for 20 min at 4°C. Ammonium sulfate was added to crude bacteriocins to reach 50% saturation for *L. acidophilus*. The solution was stimulated overnight at 4°C. Precipitates were collected by centrifugation at 10,000 g for 40 min and resuspended in 1 ml of PBS (0.05 mM, pH 7), and then, the resulting solution was divided into two tubes for concentration and desalination: one tube was transferred to a 3 kDa Amicon tube (Merck Millipore, Germany) and the second tube dialyzed against the same buffer using 12,000 kDa dialysis tubing for 48 h with 4 buffer changes [19]. The protein concentration was measured with a NanoDrop spectrophotometer (Thermo Fisher Scientific, USA). The agar well diffusion method was used to determine bacteriocin activity.

### 2.4. Statistical Analysis

The experiments were performed in triplicate under the same conditions, and the results were similar. Descriptive statistics were used to calculate the mean and standard deviation. IBM SPSS statistics software (version 25.0) was used for statistical analysis.

## 3. Results

### 3.1. Bacteriocin Production Assay in Solid Media by Overlay Soft Agar Method

In the overlay soft agar method, an antibacterial effect was observed against the standard strain of MSSA (ATCC 25923) and MRSA (ATCC 33591) (Figure 1). In the 24 h incubation period at 37°C, the diameter of the growth inhibition zones was larger than the incubation period in 48 h and 72 h for MRSA and MSSA (see Table 1). Growth inhibition was greater for MSSA than for MRSA.

### 3.2. Bacteriocin Production Assay in CFS by Agar Well Diffusion and Modification of Punch Hole Methods

No antibacterial effect was observed in neutralized CFS and not neutralized CFS of *L. acidophilus* ATCC 4356 with changes in TSB, BHI, and MRS liquid culture media for 24, 48, and 72 hours of incubation at 30°C and 37°C, against MSSA and MRSA by agar well diffusion and modification of punch hole methods.

### 3.3. Bacteriocin Production Assay in Suspension by the Paper Disk Method

No antibacterial effect was observed in the suspension of *L. acidophilus* ATCC 4356 for 24 h of incubation at 37°C, against MSSA and MRSA by the paper disk method.

### 3.4. The Concentration of Crude Bacteriocin Obtained by Ammonium Sulfate Method and Measurement of Its Antibacterial Activity

The concentration of the crude bacteriocin obtained was 22 mg/ml and 12 mg/ml. 22 mg/ml was related to desalination by ultrafiltration method, and 12 mg/ml was related to desalination using a dialysis tube. No antibacterial effect was observed in crude bacteriocin *L. acidophilus* ATCC 4356 obtained by ammonium sulfate method for 24 h of incubation at 37°C, against MSSA and MRSA by agar well diffusion.

## 4. Discussion and Conclusion

Bacteriocins are antimicrobial peptides (AMPs), and many lactic acid bacteria (LAB) can produce them. The bacteriocins used as potential therapeutic agents in the fight against infections caused by multi-drug-resistant microorganisms are interesting candidates for further development as antimicrobial agents used in health fields.

In our study, different methods were used to measure bacteriocin production and determine the antimicrobial effect of *L. acidophilus* ATCC 4356 against MSSA and MRSA. The first step and method for screening bacteriocin was overlay soft agar that was done on a solid culture medium. The next step was the use of the additional test in a liquid medium that are confirmatory methods including agar well diffusion, modification of punch hole, and paper disk method. We only observed an antibacterial effect by the overlay soft agar method in triplicate tests. The diameter of the growth inhibition zones in 24 h was larger than the incubation period in 48 h and 72 h at 37°C. In the study conducted by Pato et al. in 2021, the results were similar to our study [20]. They reported that the maximum antimicrobial activity was achieved at 24 h of incubation and then reduced from 36 h to 72 h of incubation [20]. The increase in growth inhibition zones in 24 h may be due to the growth of LAB during the 12-24-hour incubation period in the stationary phase, as secondary metabolites such as bacteriocin are formed more in this phase [20]. Some studies had different results than ours, which may be due to differences in the type of bacteriocins produced in bacteria [21, 22].

The antibacterial effect detected by the overlay soft agar method according to other studies may be due to the production of bacteriocin-like substances (BLS) that LAB are capable of producing [10]. BLS is water-suitable, active in excess of a varied range of pH values, and unaffected by lipolytic and proteolytic enzymes [10]. The expression of BLS in a liquid culture medium is very limited or nonexistent [23]. In a study, Aslim et al. showed that *L. plantarum*, *L. fermentum*, and *L. acidophilus* isolated from Turkish dairy products have inhibitory activity against *S. aureus* due to BLS production [24].

In our study, no antibacterial effect was observed in crude bacteriocin *L. acidophilus* ATCC 4356 obtained by the ammonium sulfate method. If the level of expression of bacteriocin in the liquid culture medium is low, the use of biochemical methods to obtain the purity of crude bacteriocin from the supernatant of bacteriocin-producing strains is not useful. [10]. In another study by Mobarez et al. in 2008, they reported that the antimicrobial activity of the crude bacteriocin produced in CFS by *L. acidophilus* against *Pseudomonas aeruginosa* was more than that of *S. aureus*, which indicated the limited activity of the CFS of this bacterium against *S. aureus* [25].

## 5. Conclusion

We conclude that the antibacterial effect observed by the overlay soft agar method may be due to the BLS production instead of bacteriocins. In this study, *L. acidophilus* ATCC 4356 bacteriocins had shown no or limited antibacterial activity against MSSA and MRSA. The overlay soft agar method is a qualitative test. As a result, there is a need for further study to optimize the conditions for the production of BLS in the CFS and precise comparison between the inhibitory activity and pheromone secretion of different strains.

## Figures and Tables

**Figure 1:** Bacteriocin production assay in *L. acidophilus* ATCC 4356 against MRSA by overlay soft agar method.

**Table 1:** The size of the diameter of the growth inhibition zone according to the incubation time at 37°C against MSSA and MRSA.

Incubation time period at 37°C	The size of the diameter of the growth inhibition zone (mm), mean ± SD	
	MSSA	MRSA
24 h	33 ± 2	26 ± 2.5
48 h	14 ± 1	12.6 ± 0.5
72 h	11 ± 1.5	10 ± 1

## Data Availability

All data utilized or generated in this study are displayed in tables and figures within the manuscript.
